# Attention Layer-Based Multidimensional Feature Extraction for Diagnosis of Lung Cancer

This article has been retracted.

**DOI:** 10.1155/2022/3947434

**Published:** 2022-07-04

**Authors:** Manisha Bhende, Anuradha Thakare, V. Saravanan, K. Anbazhagan, Hemant N. Patel, Ashok Kumar

**Affiliations:** ^1^Marathwada Mitra Mandal's Institute of Technology, Pune, India; ^2^Department of Computer Engineering, Pimpri Chinchwad College of Engineering, Pune, India; ^3^Dambi Dollo University, Ethiopia; ^4^Department of Computer Science and Engineering, Saveetha School of Engineering, SIMATS, Chennai, India; ^5^Computer Engineering, Sankalchand Patel College of Engineering, India; ^6^Department of Computer Science, Banasthali Vidyapith, Banasthali-304022 (Rajasthan), India

## Abstract

At present, early lung cancer screening is mainly based on radiologists' experience in diagnosing benign and malignant pulmonary nodules by lung CT images. On the other hand, intraoperative rapid freezing pathology needs to analyse the invasive adenocarcinoma nodules with the worst recovery in adenocarcinoma. Moreover, rapid freezing pathology has a low diagnostic accuracy for small-diameter nodules. Because of the above problems, an algorithm for diagnosing invasive adenocarcinoma nodules in ground-glass pulmonary nodules is based on CT images. According to the nodule space information and plane features, sample data of different dimensions are designed, namely, 3D space and 2D plane feature samples. The network structure is designed based on the attention mechanism and residual learning unit; 2D and 3D neural networks are along built. By fusing the feature vectors extracted from networks of different dimensions, the diagnosis results of invasive adenocarcinoma nodules are finally obtained. The algorithm was studied on 1760 ground-glass nodules with 5-20 mm diameter collected from a city chest hospital with surgical and pathological results. There were 340 nodules with invasive adenocarcinoma and 340 with noninvasive adenocarcinoma. A total of 1420 invasive nodule samples were cross-validated on this example dataset. The classification accuracy of the algorithm was 82.7%, the sensitivity was 82.9%, and the specificity was 82.6%.

## 1. Introduction

Lung cancer has recently emerged as a malignancy that poses a major threat to human health as one of its symptoms [1]. When opposed to other tumors, lung cancer has no symptoms in the early stages. Many patients have progressed to the point where they are inoperable or have metastasized, and patients in the middle and late stages have poor surgical outcomes [2, 3]. Lung cancer screening with low-dose helical CT is critical for early diagnosis of lung cancer, with reliable diagnostic results increasing the likelihood of a patient's capacity to be cured [4]. According to the statistics of the NLST study in the United States, in the lungs with suspected imaging in 20% of cancer cases, the final surgical pathology is not lung cancer. For lung adenocarcinoma, its subpathological type dramatically affects the surgical approach. The surgical medium-fast frozen pathology is accurate in diagnosing whether small diameter tumors are invasive, and the accuracy rate is low [5]. Therefore, for early lung cancer nodules with similar shape characteristics, the diagnosis of subpathological type of nodules, tiny nodules of lung adenocarcinoma, is based only on subjective diagnosis by radiologists which will have certain limitations and preoperative. The ability to more accurately confirm the subpathological type is also essential for the formulation of the surgical plan to have greater significance.

At present, increasing scholars are studying the use of lung CT images to perform intelligent diagnosis of pulmonary nodules to assist radiologists and improve nodules' efficiency and accuracy of diagnosis [6]. Authors have adopted a multi-input 2D convolutional net network; the input of its network is designed to contain modules, no modules, and only packets [7]. There are three different views of the same nodule object with nodule images in the common open dataset LIDC-IDRI (Lung Image Database Consortium image collection) for benign and malignant prediction of pulmonary nodules [8]. Literature medical feature parameters were extracted from CT images of 87 patients with adenocarcinoma and used different machine learning models for its invasive and noninvasive classification of gonadal carcinoma. Literature introduces center crop operation to improve the 3D DenseNet network enhancing the classification accuracy of the algorithm [9]. Literature has combined the morphological description of medical knowledge and the deep features extracted from 2D network models. Pulmonary nodules were classified using SVM (Support Vector Machine) [10]. In this study by extracting nodule morphological features and intensity characteristics to describe the nodule characteristics combined with the log, it boosts a classifier for lung cancer diagnosis [11]. Literature proposed designing a multilevel 2D cross-convolution. A residual network was utilized to predict the malignancy of the nodule [12]. Literature uses a deep residual network combined with transfer learning to compare nodular and nonnodal samples, section samples are effectively classified [13]. Literature by penetrating a comparative analysis of the lesion characteristics of adenocarcinoma and noninvasive adenocarcinoma confirmed that the average diameter and shape of the lesions could provide a good reference for the construction of diagnostic models [14]. In literature, a multidimensional convolutional neural network is designed using three-dimensional images and two-dimensional multiscale images of nodules which are trained and classified, and the two classification results of the class network are weighted and fused to classify pulmonary nodules [15]. The essential benefit of CNN over its counterparts will be that it discovers essential qualities but without human intervention. Despite a big number of photos of dogs, it can learn distinct features for each category on its own. In contrast, CNN is computationally efficient. Along with some of its drawbacks such as the location of an object are not represented by CNN [16]. Inability to be substantially invariant when coping with incoming information and it is essential to collect a high volume of data [17].

Most of the current research is to design a 2D or 3D network as a classification algorithm for pulmonary nodules alone or to use machine learning algorithms for classification based on nodule feature parameters. The fusion in multidimensional convolutional neural network of authors combines the classification results of 2D and 3D networks [18]. However, like many existing networks, only the original image information of nodules is learned, which is different from medical research. Prior knowledge is less combined. Due to the lack of datasets of pulmonary nodules, it cannot reach more than 10,000 cases like other large datasets, and fewer studies are using deep learning to classify invasive adenocarcinoma nodules and noninvasive nodules. Provide adequate diagnostic help in preoperative preparation. For author survey classification of invasive adenocarcinoma, they used the random forest method to achieve an accuracy of 86.7% with a sensitivity of 66.7% and a specificity of 100%, but the total number of samples in their study was only 87%. For example, the classification accuracy has a significant chance, and an enormous sacrifice has been made in the diagnosis accuracy of malignant samples. An elevated sensing layer relying on dual-template biochemically functional monomer was devised and extensively utilized to detect CEA and AFP as lung cancer diagnostics one at a moment. The authors have proposed the specific 3D model for lung nodule extraction of CT images which provides the learning algorithm through many sizes and integrates elements in a lowest part hierarchical manner for investigation purpose.

In our proposed study, the network design includes an attention mechanism and a residual learning module. The 2D and 3D convolutional networks are trained separately initially, followed by the extraction of the two sets of network outputs. The eigenvectors are concatenated into new eigenvectors, and the classifier is retrained with XGBoost to improve its accuracy even more. The spatial and planar features of nodules have been thoroughly investigated in our study. The results showed that the different feature vectors extracted under the dimension are fused and reclassified. The classification result is better than the results of 2D network or 3D network classification alone and can be used in the accuracy, sensitivity, and specificity which can achieve a reasonable level. Hence, in this study, we investigated invasive adenocarcinoma nodules in ground-glass nodules during surgery. The previous diagnosis, different from the public dataset LIDC-IDRI samples from the subjective judgment of the existence of multiple radiologists, is different; this paper collects from Shanghai Chest Hospital with the gold standard, that is, with postoperative pathological support 1760 CT samples of ground-glass pulmonary nodules with invasive adenocarcinoma 340 nodules and 1420 noninvasive nodules in each CT sample containing 20 CT slices with a continuous slice thickness of 1 mm. For lungs in different samples due to the significant difference in nodule size and attention mechanism-based residual differential network model, using the designed 3D convolutional network and 2D convolutional network, respectively, the network extracts different feature information, removing the features from the other dimension networks. Finally, the vectors are concatenated into a new feature vector, and XGBoost is used for training analysis. The classification and diagnosis of invasive adenocarcinoma in pulmonary nodules were finally completed.

### 1.1. Organization

The paper has been organized as follows.  Section 1 describes the introduction of the problem statement followed by Section 2 which elucidates the method description.  Section 3 talks about the application and analysis followed by Section 4 which states the conclusion obtained from the strategy.

## 2. Method Description

As shown in Figure 1, the different dimensions of the attention mechanism proposed in this paper and the degree of network extraction feature fusion model AFCNN (Attention Fusion, implementation of Convolutional Neural Network) are mainly divided into the following: image preprocessing, data enhancement, and classifier structure construction.

The original dataset is an image preprocessed to generate good 2D and 3D images; the initial dataset was used for classification of 2D data to represent lung nodule center information such as texture features and contour features of layers and 3D data to express lung nodules. All the steps are depicted in Figure 1, where the various aspects of the attention mechanism have been presented, as well as the degree of network extraction feature fusion model AFCNN, which are largely split into the following parts such as picture preprocessing where preprocessed feature extraction of images is being done followed by data augmentation, and the creation of a classifier structure construction has been represented.

Spatial feature information of CT images uses 2D data for random plane cropping, rotation, 2D cutmix, and other data enhancement methods. 3D data is spatially randomized. Data enhancement methods for extraction of spatial feature information of CT images are being employed which include cropping, spatial flipping, 3D cutmix, etc. and are being generated with 2D and 3D datasets which were trained by the network; using the proposed fusion combined model for classification, all these methods are used for preprocessing the image features to investigate lung nodule internal information in order to predict certain ailments if any. The AFCNN fusing framework has two parts: 2D ACNN (2D Attention Convolutional Neural Network) for training to extract feature vectors from 2D datasets and 3D ACNN for training to extract feature vectors from 3D datasets; the framework is being used to extract 2D features. The vectors and 3D feature vectors are converted to one-dimensional vectors and coupled to create a new feature vector that fully expresses the spatial and plane feature information of pulmonary nodules. Then, the XGBoost algorithm is used for training classification, with more accurate classification results.

### 2.1. Image Preprocessing and Data Enhancement

#### 2.1.1. Image Preprocessing

Image preprocessing on the original CT dataset is shown in Figure 2; there are two main parts: lung parenchyma extraction and lung nodule data extraction.

The lung parenchyma is extracted because the lung parenchyma is removed from the lung CT image. In addition, there is also information such as the thorax and ribs. The pixel information of these positions is for the pathological nature of pulmonary nodules and has no effect but will affect the study of nodule characteristics. Learning to cause interference and extracting lung parenchyma can strengthen the network with valuable learning features. Lung parenchyma extraction is mainly based on different pixel values in different parts to get a rough lung parenchyma outline using the threshold method to extract the lung parenchyma roughly. Then, use morphological operations and other practices to make up for the location in the lungs. In lung nodules with incorrectly cropped parenchymal margins for more accurate lung parenchyma round the contour, the contour information was used to obtain the lung parenchyma from the original CT image points and remove redundant information such as the thorax.

Pulmonary nodule data extraction uses CT images extracted from the lung parenchyma. Generate 3D image data and 2D feature image counts for each lung nodule sample according to the location information used to remove pulmonary nodules which were obtained by manual annotation. Tightly frame the nodule on the CT slice where the geometric center of the nodule is located position, mark the part of the central slice, and record the contiguous CT slice occupied by the nodule layers to mark.

Take the marked nodule center layer as the center, according to the marked nodule center layer nodule position box, and then, take the thin layers of the CT image before and after the central layer, align the crop and stitch into 3D data of size *Nx* × *Ny* × *Nz*; Nx and Ny represent the number of pixels on the CT image in the dataset. *Nz* denotes the number of CT slices, the size of which is instantiated as 32 × 32 × 9 in this study. 3D image data is used to express the spatial image information of the nodule and its surroundings. The 2D feature image data is generated from the nodule central layer image, which contains components: nodule central layer image, LBP (Local Binary Patterns), feature image, and contour feature image. 2D feature images are not in the depth direction; it is position invariant. The nodule center layer image in the component image is consistent with the image of the 3D data center layer; in this case, the image is 32 × 32 in size and converted to grayscale. The LBP feature image is mainly used to express the texture information of lung nodules, centered at each pixel; the value of the pixel covered by the window is compared with the value of the center point, according to the value of the center point and surrounding points' small relation to represent the value of the center pixel, as shown in

(1) $$\begin{array}{c} \text{LBP}\left(x_{0},y_{0}\right)=\overset{n}{\underset{i=0}{\sum }}\varepsilon \left(v_{0}-v_{i}\right)2^{i},\varepsilon \left(t\right)=\left\{\begin{array}{c} 0,t>0,\\ 1,t\leq 0. \end{array}\right. \end{array}$$

Among them, LBP (*x*_0_, *y*_0_), represents the LBP eigenvalue calculated at this point, *n* indicates the number of pixels covered by the edge of the window, which is taken as 8 in this example, *v*_*i*_ and *v*_0_ represent the pixel value of the center point and the center of the edge pixel of the *i*-th window, respectively.

The contour feature image is used to express the contour information of the nodule. In the CT image, the edges of ground-glass nodules are blurred, and operations such as Gaussian filtering are not required to work; directly use the Sobel operator to calculate the gradient of each position, to represent information on the borders of lung nodules. Each component image of the 2D feature image is, according to the image generation of the central layer of the nodule, its corresponding actual CT image. The position information is the same, and the size is *Nx* × *Ny*, in the example of this paper 32 × 32.

#### 2.1.2. Data Augmentation

Common data with respective dimensions for 2D and 3D dataset augmentation methods as well as the cut mix algorithm. Common data augmentation methods can be used, for example: image rotation in plane direction (such as 90°, 180°, and 270°), plane transpose in the direction, add Gaussian noise, etc. In particular for 2D data random cropping on the row plane, in-space random cropping of 3D data, clipping, and flipping up and down in the depth direction, enhances 2D and 3D data. The generalization performance of the set supports the training of the classifier network parameters. Due to medical, image sample collection cost is high, and the cut mix algorithm is also used in this example. Enhance the learning ability of the network for local features of lung nodules. The algorithm is right, part of the data in the sample is randomly cropped, another sample is randomly taken, and the corresponding data part is combined with the remaining part of the original sample to form a new sample, the label of the new sample is in the data of the new sample according to the two sets of samples. The proportion of the heart is combined. 2Dcutmix on the 2D dataset, i.e., perform random cropping and samples at any position and two-dimensional size on the plane fusion, perform 3Dcutmix on 3D data, that is, perform arbitrary random cropping of positions and arbitrary 3D sizes and sample fusion pass the feature fusion of different dimensions is performed on the original data, which improves the sample quality. Diversity and can enhance the ability of networks of different dimensions to local feature study.

### 2.2. Network Classifier with Attention Mechanism and Classification Training

#### 2.2.1. Design of Residual Learning Module with Attention Mechanism

The pathological diagnosis of pulmonary nodules is mainly based on partial images of pulmonary nodules, while information such as other lung parenchyma contributes to the pathological diagnosis. For ground-glass hyaluronic nodules, the proportion of images of pulmonary nodules in the acquired data sample images; the size of pulmonary nodules in different samples varies greatly. Book diameter of ground-glass pulmonary nodules in the study varied widely, which may be helpful for 5 mm to 20 mm. Due to the pixel size in CT images and the real, physical size of the lung in the physical space has a unique correspondence, and the lung scaling nodules will destroy the correspondence between the image and the physical size, loss of actual size information of lung nodules. For lung nodules of different sizes in the nodule samples, the classification of the network can be more based on the lung nodule part image information, and less reference to the image information of the lung parenchyma, so to introduce the attention mechanism when designing the network module, that is, through different channels comparison of the expression intensity of the feature images, according to the expression intensity of the feature images different to assign the corresponding feature weight to the channel.

As shown in Figure 3, a residual learning module with attention mechanism is designed. Leveraging the attention mechanism to learn to optimize the feature maps in the network during the training phase, the weight of each channel can learn the characteristics of the image that are important for classification feature, to extract important image features in the test set. This mechanism can make the network pay more attention to the information of the lung nodules, thereby improving the network classification ability of the network on this dataset. To reduce the network depth due to excessive gradient caused by the large disappears, and the residual learning module is designed to better combine the image features extracted make the extracted feature images more good participation in network classification.

In the residual learning module with attention mechanism as shown in Figure 3, the convolution transformation part consists of a convolution layer and a ReLU layer, which are used to extract the upper network feature images with the output, while the shortcut connections are made by convolution of size 1 layer composition, directly connecting the output with the upper layer network, so that the high-dimensional feature image combines better with low-dimensional feature images. The attention mechanism can be used to strengthen the weight of the important features in the convolutional transformation part.

Weight calculation of different feature channels for the attention mechanism in the module, it consists of two parts, which are the mean value and the maximum value of the characteristic images of each channel value. Let *X*_*i*_ denote the set of values of the feature image on channel *i*; then, the realization of the attention mechanism can be expressed by

(2) $$\begin{array}{c} X_{i\text{new}}=\left\{f_{1}\left[\max\left(X_{i}\right)\right]+f_{2}\left[\text{avg}\left(X_{i}\right)\right]\right\}X_{i}. \end{array}$$

Among them, *X*_*i*new_ represents the set of weighted feature images on channel *i*, max represents the maximum value in the feature image, avg represents the average value of the feature image mean, *f*_1_ represents the convolution transformation and activation function ReLU with a convolution kernel of 1 transformation combination which is Conv(1 × 1) − ReLU, the convolution with the convolution kernel of 1 the operation is used to integrate the weight information on different channels, ReLU's the effect is to enhance the nonlinearity in the attention transition. *f*_2_*s* is and the same convolutional transform structure as *f*_1_, *f*_2_, and *f*_1_ are trained separately. *f*_1_ is according to the feature image processed by the maximum value, the corresponding value of different channels is determined. Weight *f*_2_ is determined according to the average value of the processed feature images which are the corresponding weights of the channel. The weights obtained after training the two sets of attention mechanisms, results are added together, and different weights are attached to each channel of the feature image, through training, important feature channels can have greater weights, learning important features of classification significance in the image.

The essence of this mechanism is the convolutional transformation part of the module. First, each feature channel is weighted, and through the training of the above weights, the feature image with a more apparent feature expression is obtained, as shown in

(3) $$\begin{array}{c} X=\overset{c}{\underset{i=1}{\sum }}X_{i\text{new}}, \end{array}$$

where *c* is the number of channels of the feature map and *X* is the feature map of each track, like the output total feature image after the weight coefficients are superimposed.

After the feature image after the convolution transformation is weighted, the shortcut connection part uses a convolution transformation with a convolution kernel of 1 to integrate information. Finally, the divided feature images are superimposed to better integrate low-dimensional and high-dimensional features. The signature information is provided as the output of this module to the following parts of the network for training to learn.

#### 2.2.2. 2D ACNN Network Structure

2D ACNN is used to learn the plane features of lung nodules, such as edge features and texture features. The network model is designed based on the residual learning module with an attention mechanism. The detailed structure is shown in Figure 4. The network contains three residual learning modules with an attention mechanism, where Conv2D is represented by the convolutional layer, batch normalization layer, and activation layer, that is, the composite operation of Conv(*k*_*s*_ × *k*_*s*_)-BN-ReLU, where ks represents the purpose of adding batch normalisation to the size of the convolution kernel is to make the input of the activation function conform to its numerical sensitive range, thereby reducing the phenomenon of gradient disappearance, increasing the convergence ability of the network, and speeding up the training of network parameters. Avg-Max attention represents the attention mentioned above module realized by the average value and the maximum value, that is, on each channel. The relationship between input and output is Out_*i*_ = {*f*_1_[max(*X*_*i*_)] + *f*_2_[avg(*X*_*i*_)]}In_*i*_. The subscript *i* represents the component of the feature image on the *i*-th channel; in the 2D network, the feature component is two-dimensional, and the transformation is denoted as *g*. With the attention machine, the output of the residual learning module is controlled by the attention module, and the convolution kernel is 1. The block outputs are added together, i.e., *X*_out_ = *g*(*X*_in_) + *h*(*X*_in_), *X*_in_ is the input of this learning module, and *X*_in_ is the input of the attention module by *X*_in_. After two Conv2D module operations, *h* represents the convolution kernel with 1 Conv2D transformation. The convolution kernel setting for the input layer Conv2D of this network is 7; to increase the receptive field of the upper layer of the network, MaxPool means the most. A large pooling operation reduces the number of parameters the network needs to train. Adaptive Avg Pool represents a global average pooling operation for each channel. The feature images are globally pooled, and the average value is used to describe the channel's eigenvalues. Output the 2D feature vector after global pooling, through the full convolution linear layer for classification.

#### 2.2.3. 3DACNN Network Structure

3D ACNN is used to learn the spatial information of pulmonary nodules. The Spatial features are invariant in the depth direction, so the 3D network structure is designed to the structure to understand contextual information from lung nodule data. To reduce network requirements with the number of parameters to be trained, the network model mainly has three machines' attention. The detailed structure of the residual learning module is shown in Figure 5. Conv3D representation is implemented by a convolutional layer, batch normalization layer, and activation layer, namely, Conv (*k*_*s*_ × *k*_*s*_ × *k*_*s*_)—composite operation of BN-ReLU, where *k*_*s*_ represents the volume in this case, the size of the kernel, the length, width, and depth of the kernel. The size remains the same; Avg-Max attention is the average and maximum value. The current attention module is Out_*i*_ = {*f*_1_[max(*X*_*i*_)] + *f*_2_[avg(*X*_*i*_)]}In_*i*_. In a 3D network, the feature components on channel *i* are three-dimensional, and the transformation is denoted by *a* for *g*. The output of the residual learning module with the attention mechanism is *X*_out_ = *g*(*X*_in_) + *h*(*X*_in_), where *X*_in_ passed through the Conv3D module twice by *X*_in_. The operation is obtained; *h* represents the Conv3D transform with a convolution kernel of 1 in the network.

The convolution kernels of the Conv3D are all set to 3, reducing the need for training the network—the number of parameters to exercise. Adaptive AvgPool represents the global average pooling operation to global pooling on the 3D feature images on each channel, using the flat mean to represent the eigenvalues of the channel. Output 3D features after the global pooling *A* vector is classified by a fully convolutional linear layer.

#### 2.2.4. Classification Objective Function and Feature Fusion

The 2D network and 3D network are trained separately, and the goal of network optimization is to minimize the loss function. Because of the binary classification problem to be solved in the research, the loss function is selected as a binary cross-entropy function, and a regularization term is added, as shown in

(4) $$\begin{array}{c} \text{Loss}=-\frac{1}{n}\overset{n}{\underset{i=1}{\sum }}\left(y_{i}\ln y_{e}+\left(1-y_{i}\right)\ln\left(1-y_{e}\right)\right)+\alpha \sum {\left\|w_{i}\right\|}_{2}^{2}. \end{array}$$

Among them, *y*_*i*_ is the label of sample *i*, *y*_*e*_ is the classifier's prediction for the sample *i* label, *n* is the total number of samples, *α*∑‖*w*_*i*_‖_2_^2^ is the regularisation term, and *α* is positive. The normalisation coefficient is generally a small positive number, and ‖*w*_*i*_‖^2^ is the weight coefficient in the network, which is the second norm of a number. L2 regularization controls the value of the objective function by optimizing the size of the weight parameters in the network, reducing the complexity of the network, and reducing the network overload fit.

After the two groups of networks are trained separately, take the output of the 2D network in Figure 4. The 2D feature vector and the 3D feature vector output by the 3D network in line feature fusion, because the 2D feature vector and the 3D feature vector are the corresponding feature vector extracted by the network for binary classification so that it can express 3D spatial features and 2D plane features, the implementation method of feature fusion is to combine the network. The 2D feature vector and 3D feature vector output by the network are converted into one-dimensional amount make the connection, that is *v*_new_ = [*v*_3*D*_^1^, *v*_3*D*_^2^, *v*_3*D*_^3^⋯, *v*_3*D*_^*k*^, *v*_2*D*_^1^, *v*_2*D*_^2^, ⋯, *v*_2*D*_^*k*^], where *v*_3*D*_^1^ represents the vector of the 1st channel in the 3D feature vector and the *v*_2*D*_^1^ table shows the vector of the 1st channel in the 2D feature vector. Therefore, *k* represents the total number of channels of the 3D feature vector, and *t* is the total number of channels of the 2D feature vector number. Take new as the new feature vector of the sample and use XGBoost to calculate the method to classify and learn the new feature vector; the obtained classification result is the final classification result of this classifier. In the experiment, XGBoost chooses every. The second tree-based model is iterated, the iteration weight eta is designed to be 0.1, and the tree. The maximum depth of 5 is designed to avoid overfitting, the goal of the XGBoost model. The optimization function is consistent with formula (4).

## 3. Example Application and Analysis

The datasets used in this paper are from Shanghai Chest Hospital all over the years. Cases with accurate pathology after surgery, between 5 mm and 20 mm in diameter ground-glass pulmonary nodule samples a total of 1760 cases, invasive 340 samples of adenocarcinoma nodules and 1420 samples of noninvasive adenocarcinoma nodules examples. In noninvasive nodule samples microinvasive adenocarcinoma, primary adenocarcinoma, and other benign nodules each case data contains a slice thickness of 20 consecutive CT thin-slice images of 1 mm. Compared to most research papers, the LIDC-IDRI public dataset of this research, the dataset of this research has the gold standard, the public dataset of benign and malignant nodule samples was determined by four radiologists. The doctors independently marked the pulmonary nodules into five grades from 1 to 5 according to the degree of malignancy, with 5 representing the highest degree of malignancy and 1 representing a benign nodule. However, the doctor's diagnosis is subjective; in the diagnosis of 1 187 cases of nodules, four doctors, only 571 nodules were diagnosed as valid if the difference between the judging results of the judging results was less than 1. Unfortunately, the difference between the diagnoses of different doctors in the rest of the samples was large. Therefore, the annotation of the public dataset cannot be used as actual pulmonary nodule pathology, and the dataset contains different types of nodules, such as ground-glass nodules and solid nodules—classification of invasive adenocarcinoma.

The configuration of the experimental platform running in this article is an Intel Core i9-9900 processor, NVIDIA GeForce RTX 2080Ti discrete graphics card, and 32 GB memory. The experiment's data processing and model building are based on the thepython3.7, mainly based on PyTorch's deep learning framework. In the experiment, the parameters in the network are initialized using the Keming method.

The proposed algorithm was verified using five-fold cross-validation to make the network thoroughly trained and reduce the training results by chance. The original dataset was randomly divided into five independent parts of the same size. Sixty-eight samples contained invasive adenocarcinoma nodules and noninvasive adenocarcinoma 284 cancer nodules samples. In the *i*-th verification, select the *i*-th sample as the test set, the remaining four samples are used as the training set for training, that is, each activity. The ratio of the training set to test set in practice is 4 : 1. Initial training set: A total of 1 408 samples were collected, including 272 invasive adenocarcinoma nodules and 272 noninvasive adenocarcinoma nodules. One thousand one hundred thirty-six samples of invasive adenocarcinoma nodules. Data augmentation during training Strong augmented the training set to 84 224, in which invasive adenocarcinoma samples and noninvasive adenocarcinoma samples were 1 : 1.

Five experiments were conducted to train and verify the two networks, respectively. Record the results, fuse the training results of the two networks, and record their development. The size of the 2D samples in the experiment is instantiated as 32 × 32, and the 3D sample size of a is instantiated as 32 × 32 × 9, the regularization coefficient *α* is taken as 0.000 01; in this paper, the SGD optimizer is used for optimization, and the initial learning of the training network is the learning rate is designed to be 0.02, the momentum parameter is set to 0.9, and the learning rate is set to 10 times line attenuation. The selection of the initial learning rate is based on the experimental results in Table 1.

In network training, it will not be easy to converge if the learning rate is set too high. On the other hand, if the habit rate is too low, it will be trapped in local maxima. In this experiment, according to the table the results in 1 show that when the initial learning rate is 0.02, it can be achieved without sacrificing sensitivity and specificity and have higher accuracy, so the initial learning rate in this order of magnitude is 0.02. The regularization coefficient should not be too high large; it will hinder network training, so taking a smaller value of 10E−5 can prevent overfitting. However, it plays a specific limiting role, and the fluctuation of this value will affect the experimental results with little noise.

This experiment used three accuracies, sensitivity, and specificity methods, respectively. Metrics evaluate the performance of the model. The definition of the indicator is shown in [18]

(5) $$\begin{array}{c} \left\{\begin{array}{c} \text{Accuracy}=\frac{\text{TP}+\text{TN}}{\text{TP}+\text{TN}+\text{FP}+\text{FN}},\\ \text{Sensitivity}=\frac{\text{TP}}{\text{TP}+\text{FN}},\\ \text{Specificity}=\frac{\text{TN}}{\text{TN}+\text{FP}}. \end{array}\right. \end{array}$$

Among them, TP represents the sample whose correct category and prediction result are positive quantities. TN means the number of pieces whose right category and predicted result are negative quantities. FP represents the number of samples whose actual class is negative and expected to be positive. FN indicates the number of samples where the actual class is positive, and the prediction is negative. In this instance, the sensitivity indicates that the class of invasive adenocarcinoma is correctly predicted. The specificity represents the proportion of samples classified as noninvasive predicting the correct proportion [18].

As shown in Figure 6, some lung nodules on the test set are classified by the model in this paper—class error visualization results—box-select three of the noninvasive adenocarcinoma nodules. The actual pathology of the nodules in the group was noninvasive, but they were diagnosed as invasive nodules. The corresponding percentages are the probability of a diagnosis of an invasive nodule. Boxed in dip the actual pathology of the three groups of nodules of invasive adenocarcinoma was invasive nodules. Still, the model, probability of predicting it as an invasive nodule is shallow, so the final classification the result is a noninvasive nodule. In the figure, the similarity between the two groups of pulmonary nodules is very high. The first two groups of nodules in invasive adenocarcinoma were regular in shape. They had regular density value and rhythm, while the noninvasive clusters of nodules were irregular in shape, leading to type produced misjudgment.

The results of the five-fold cross-validation are shown in Figure 7, which, respectively, represent the five experimental groups. The accuracy sensitivity and specificity of the test results, the Abscissa in the graph both represents the experimental group number, and the ordinate represents the accuracy and sensitivity values, respectively. Specificity values, the three curves in each graph represent the 3D network classification results, 2D network classification results alone, and the classification result after feature fusion. For example, Figure 7(a) shows the three methods in five accuracy results on the group test set; 2d networks generally perform across groups. Poor, with an average accuracy of 0.753, the 3D network outperformed each group's 2D network with an average accuracy of 0.814; since the 3D dataset has more, the dataset is more informative, and the spatial characteristics of the modules are more effective for the classification results. Flat features have a more substantial effect. The fusion classification result combines 2D network, the extracted feature vectors, and the feature vectors extracted by the 3D network, so you can combine spatial features and plane features to get better classification accuracy, the average. The accuracy is 0.827.  Figure 7(b) shows the sensitivity results of the three methods results, classification results of 2D network and 3D network on different sets of datasets.

There is no clear distinction between superiority and inferiority, as sensitivity is shown in invasive adenocarcinoma. The raw data volume is small when it is diagnosed with the correct scale, so the 2D network is similar. There is no noticeable difference in the classification results of the 3D network [3, 19]. The fusion classification is after spatial features and planar features; there is no improvement in the fourth set of experiments [1, 20]. The rest, sensitivity of fusion classification in the group, has been dramatically improved.  Figure 7(c) shows the specificity results of the three methods were compared, and the specificity of the 2D network was significantly lower than 3D networks, which is consistent with the experimental results on the accuracy; the 3D network can learn more information by merging features of different dimensions, it can make the specificity been improved to a certain extent.  Table 2 shows the accuracy, sensitivity, and specificity of five-fold cross-validation.

The study of the classification of invasive adenocarcinoma in this paper is based on the gold standard. A total of 1 187 samples were obtained. To compare the manual diagnosis of invasive adenocarcinoma nodules, 20 samples were randomly selected from the dataset, and one a doctor with many years of experience made a diagnosis. The doctor's diagnosis accuracy is 70%. As shown in Figure 7, the algorithm's accuracy proposed in this paper is 0.827, the sensitivity was 0.829, and the specificity was 0.826. Visible relative to physician experience, it can be concluded that the method in this paper can significantly improve the misdiagnosis rate in the diagnosis of invasive adenocarcinoma nodules and noninvasive nodules. It shows that the model in this paper can pass the pulmonary nodules. It can learn the image information of nodules and obtain good diagnostic ability of invasive nodules High accuracy without sacrificing classification sensitivity and specificity.

## 4. Conclusion

Small nodules in invasive adenocarcinoma could well be diagnosed using the proposed method in this research. In this approach the attention process supports the multidimensional and multifeature fusion classification model; initially, lung parenchyma was extracted from the original CT picture to remove interfering information like thorax interest. The 2D lung nodule samples in the output of the model in the design are central layer images, LBP features, and round, to improve the model's learning of lung nodule features. The 3D lung nodule sample is made up of many CT slices. In this study the application of traditional data enhancement methods and the cut-mix algorithm to enhance the generalizability of the dataset can improve the ability of the network to learn valuable features for pulmonary nodules on the web, given the characteristics of the dataset, which include a small sample size and unbalanced samples. The network design includes an attention mechanism and a residual learning module. The 2D and 3D convolutional networks are trained separately initially, followed by the extraction of the two sets of network outputs. The eigenvectors are concatenated into new eigenvectors, and the classifier is retrained with XGBoost to improve its accuracy even more. The spatial and planar features of nodules have been thoroughly investigated in our study. The results showed that the different feature vector extracted under the dimension is fused and reclassified. The classification result is better than the results of 2D network or 3D network classification alone and can be used in the accuracy, sensitivity, and specificity can achieve a reasonable level. The technique was applied to nodules with a diameter of 5-20 mm that were gathered from Shanghai Chest Hospital. There were 340 invasive adenocarcinoma nodule samples and 1420 noninvasive adenocarcinoma samples. The nodule samples were examined, and cross-validation revealed that the classification accuracy was 82.7%, the sensitivity was 82.9%, and the specificity was 82.6%. The purpose of this paper is to classify and evaluate subpathological forms of ground-glass nodules, as well as to provide additional practical information algorithms for diagnosis.

## Figures and Tables

**Figure 1:** Model implementation process.

**Figure 2:** Image preprocessing.

**Figure 3:** Network module with attention mechanism.

**Figure 4:** 2D ACNN network structure.

**Figure 5:** 3D ACNN network structure.

**Figure 6:** Some samples of the wrong classification of the model.

**Figure 7:** Accuracy, sensitivity, and specificity of five-fold cross-validation.

**Table 1:** Experimental result of 2D and 3D networks with different learning rates.

Learning rate	Accuracy		Sensitivity		Specificity	
	2D	3D	2D	3D	2D	3D
0.3	0.844	0.904	0.835	0.889	0.846	0.91
0.03	0.85	0.921	0.889	0.909	0.843	0.924
0.003	0.722	0.927	0.835	0.85	0.818	0.945

**(a):** 

Group no.	3D network classification results	2D network classification results	Fusion classification results
1	0.75	0.825	0.885
2	0.78	0.858	0.9204
3	0.74	0.814	0.8732
4	0.72	0.792	0.8496
5	0.8	0.88	0.944

**(b):** 

Group no.	3D network classification results	2D network classification results	Fusion classification results
1	0.75	0.87	0.9
2	0.78	0.9048	0.936
3	0.74	0.8584	0.888
4	0.72	0.8352	0.864
5	0.8	0.928	0.96

**(c):** 

Group no.	3D network classification results	2D network classification results	Fusion classification results
1	0.75	0.87	0.93
2	0.78	0.9048	0.9672
3	0.74	0.8584	0.9176
4	0.72	0.8352	0.8928
5	0.8	0.928	0.992

## Data Availability

The data shall be made available on request.
